# Modeling the Impact of Seasonal Weather Variations on the Infectiology of Brucellosis

**DOI:** 10.1155/2020/8972063

**Published:** 2020-10-17

**Authors:** Nkuba Nyerere, Livingstone S. Luboobi, Saul C. Mpeshe, Gabriel M. Shirima

**Affiliations:** ^1^Department of Applied Mathematics and Computational Sciences, Nelson Mandela African Institution of Science and Technology, P.O. Box 447, Arusha, Tanzania; ^2^Department of Mathematics, Informatics and Computational Sciences, Sokoine University of Agriculture, P.O. Box 3038, Morogoro, Tanzania; ^3^Institute of Mathematical Sciences, Strathmore University, P.O. Box 59857-00200, Nairobi, Kenya; ^4^Department of Mathematics, University of Iringa, P.O. Box 200, Iringa, Tanzania; ^5^Department of Global Health and Bio-Medical Sciences, Nelson Mandela African Institution of Science and Technology, P.O. Box 447, Arusha, Tanzania

## Abstract

A deterministic mathematical model for brucellosis that incorporates seasonality on direct and indirect transmission parameters for domestic ruminants, wild animals, humans, and the environment was formulated and analyzed in this paper. Both analytical and numerical simulations are presented. From this study, the findings show that variations in seasonal weather have the great impact on the transmission dynamics of brucellosis in humans, livestock, and wild animals. Thus, in order for the disease to be controlled or eliminated, measures should be timely implemented upon the fluctuation in the transmission of the disease.

## 1. Introduction

Brucellosis is a bacterial zoonosis that causes potential loss of production in livestock and undulant fever in humans in many countries all over the world [1]. The infection is caused by the genus *Brucella* with *B. melitensis*, *B. suis*, and *B. abortus* being predominant in domestic animals and also infecting humans [2–4]. International organizations like the World Organisation for Animal Health (Office International des Epizooties (OIE)), the World Health Organization (WHO), and the Food and Agriculture Organization (FAO) identify brucellosis as one of the most prevalent zoonoses in the world alongside bovine tuberculosis and rabies [5].

In most parts of the developing world, brucellosis is endemic and leads to devastating losses in the livestock industry especially to smallholder keepers and to international market [6]. The disease results in huge financial losses by causing abortions, sterility, decreased milk production, veterinary fees, and cost of replacing animals. In many countries of sub-Saharan Africa, the control of the disease had proven to be a challenge because of different farming systems, low community awareness about the disease, poor health network systems, weak surveillance programmes, and limited vaccinations [7]. In animals, brucellosis is transmitted when a susceptible animal ingests contaminated materials such as pastures or discharges from infected animals while in humans, the bacteria are transmitted through ingestion of contaminated raw blood, meat, dairy products, and unpasteurized milk. Brucellosis is an occupational disease to abattoir workers, farmers, veterinarians, and laboratory personnel through direct contact with aborted materials and discharges, handling of suspected samples, and handling of livestock during deliveries [8]. Although traditionally *Brucella* species are host specific, recent studies revealed that cattle are also susceptible to *B. melitensis* [9–11].

Infected animals exhibit clinical signs like reduced fertility, late-term abortion, considerable drop in milk production, retained placenta, metritis, and hygromas in chronic cases in cattle [6, 12]. Symptoms in humans include headache, weakness, continuous or intermittent fever, chills, joint pains, profuse sweats, weight loss, aches, and devastating complications that may lead to miscarriage during the first trimester in pregnant women. Endocarditis, bone abscesses, or testicular and neurological complications can also occur [1, 13]. Human brucellosis is debilitating and needs prolonged treatment using a combination of antibiotics [14]. Furthermore, the clinical signs of the disease in humans are not pathognomonic; hence, patients were clinically misdiagnosed with malaria, rheumatic fever, typhoid fever, elapsing fever, and joint diseases [15].

Globally, the burden of human brucellosis remains huge; more than 500,000 new cases per year are reported [8]. Brucellosis exists throughout the sub-Saharan African region, it is poorly understood with fluctuating records from one country to another, and its prevalence is still unclear [16]. In many parts of Tanzania, brucellosis is a highly prevalent disease. However, very limited data is available regarding its distribution, affected host species, and impact. In addition, it has been demonstrated that the cattle seroprevalence level in various production systems, zones, and regions varies from 1 to 30% while in humans, the average prevalence is from 1 to 5% [17]. A study by Carugati et al. [18] shows that brucellosis incidences are moderate in the northern part of Tanzania and that it is a common human health problem since it is endemic in the region. Human brucellosis cases have also been reported in parts of eastern, lake, and western regions of Tanzania with seroprevalences varying from 0.7 to 20.5% [19, 20].

The incidence and prevalence of most infectious diseases are directly linked to seasonal weather variations. The understanding of seasonal patterns in infectious disease occurrences dates back to the Hippocratic era [21]. The seasonal weather variations influence the dynamics of infectious diseases by affecting the host-pathogen interactions which alters the components of the reproduction number [22]. In particular, cold or wet seasons are associated with high disease incidences due to the abundance, survival, and virulence of pathogens and the fact that most people spend their time in poorly ventilated houses. On the other hand, warm or dry seasons are associated with decreased disease incidences due to increased outdoor activities and exposure of the pathogens to UV light. In addition, the survival of pathogens outside their hosts depends on other environmental factors such as humidity, salinity, temperature, and soil pH, abundance of vectors and nonhuman hosts, host immune function, and host behavior [23].

Mathematical models can give insight into how the mechanisms and strength of seasonality affect the persistence and spreading of communicable diseases. In this view, understanding the impact of seasonality and timing offers important intuitions on parasite-host system operation, how and when the parasite control measures should be applied, and the response of disease risks to anthropogenic climate change and patterns of seasonality.

Seasonal variations are exhibited in brucellosis incidences where a large number of new cases are expected in months with wet or dry seasons of the year in both developing and developed countries [19]. The disease incidence is higher during the wet season; breeding is synchronized for animals to give birth during the wet season when pastures are available. Pastoral and agropastoral settings depend on natural pastures. During this time, infected animals shed pathogens into the environment through birth fluids and tissues that contaminate pastures and the surroundings. In addition, during the wet season, it is anticipated that the cold weather favours survival of *Brucella* pathogens in the environment compared to the hot dry season hence influencing the transmission rate [24]. For instance, high transmission rates between domestic and wild animals are expected during the dry season due to sharing of pastures and water points, while the within-herd transmission is expected during the wet season due to a high birth rate and abortion storms [25]. According to the WHO [8], in countries with cold or temperate climates, there are notable seasonal variations in brucellosis incidences with most occurring cases in the summer and spring. This concurs with the peak period for parturitions and abortions in animals and consequently the highest level of exposure to other animals and people consuming their products or attending the animals. Seasonality in transmission dynamics of the disease is also attributed to seasonal livestock movements due to the availability of water and grasslands. This is the common practice in sub-Saharan Africa countries; for instance, during the dry seasons, 83.1% of the cattle owners in Northern Tanzania move their cattle away from homes for pasture and water needs [25]. This changes the disease dynamics since the concentration of animals is expected near water bodies and wildlife parks and increases the contact rates between susceptible and infected animals.

*Brucella* is a robust pathogen, and it can persevere outside and inside the mammalian hosts for a long time despite the unfriendly conditions; it remains in food for up to 15 months given adverse conditions such as acidity and temperature between 14°C and 11°C or for two to three days under 37°C. When *Brucella* is exposed directly to sunlight, it may survive for few hours while its survival in contaminated manure and aborted foeti is more than 2 months during the winter season [26]. Furthermore, in an ideal environment, the survival of *Brucella* spp. is reported to last up to 135 days [27]. Therefore, to estimate the impact of seasonality on brucellosis transmission in animals and humans using mathematical modeling becomes imperative to device timely interventions. Despite the fact that the WHO, FAO, and OIE efforts and interventions are available, brucellosis continues to pose great economic threats and it affects livelihoods and food security mostly in developing countries. Thus, there is need to assess the impact of the current control strategies if we are to control or eradicate the disease. So far, a few studies [28–34] analyzed the dynamics and spread of brucellosis in homogeneous/heterogeneous populations. However, none of these studies have considered the mathematical approach to analyze the impact of seasonal weather variations on the transmission of brucellosis in human, livestock, and wildlife populations. In this paper, the impacts of seasonal weather parameters on the transmission of brucellosis are studied using a mathematical model.

## 2. Model Formulation

A deterministic mathematical model that illustrates the transmission of brucellosis in humans and domestic and wild animals is formulated and analyzed under this section. More importantly, in incorporating the variations on seasonal weather in both direct and indirect transmission routes of the disease, we follow the approach presented in [33, 35, 36]. The stimuli of seasonal variations on the direct transmission of brucellosis in domestic ruminants, humans, and wild animals are, respectively, modeled by the periodic continuous functions *β*_a_(*t*) = *b*_1_(1 + *a*_1_sin*ωt*), *β*_h_(*t*) = *b*_2_(1 + *a*_2_sin*ωt*), and *β*_w_(*t*) = *b*_3_(1 + *a*_3_sin*ωt*) while the indirect transmission in the three populations is captured by *α*_a_(*t*) = *c*_1_(1 + *r*_1_sin*ωt*), *α*_h_(*t*) = *c*_2_(1 + *r*_2_sin*ωt*), and *α*_w_(*t*) = *c*_3_(1 + *r*_3_sin*ωt*), respectively.

Furthermore, we consider the pathogen shedding rate by the infective livestock and wild animals to be represented by the periodic functions of the form *ρ*(*t*) = *ρ*_0_(1 + *ρ*_1_sin*ωt*) and *ρ*_w_(*t*) = *ρ*_2_(1 + *ρ*_3_sin*ωt*), respectively. The decaying rate of the pathogens in the environment is also represented by the periodic continuous function *ε*(*t*) = *ε*_0_(1 + *ε*_1_sin*ωt*). The constants *b*_1_, *b*_2_, *b*_3_, *c*_1_, *c*_2_, *c*_3_, *ρ*_0_, *ρ*_2_, and *ε*_0_ are the baseline values of the parameters *β*_a_, *β*_h_, *β*_w_, *α*_a_, *α*_h_, *α*_w_, *ρ*_a_, *ρ*_w_, and *ε*, respectively, whereas 0 < *a*_1_, *a*_2_, *a*_3_, *r*_1_, *r*_2_, *r*_3_, *ρ*_1_, *ρ*_3_, *ε*_1_ < 1 are the strength of seasonal forcing in transmission (amplitudes of seasonal variations) for each of the seasonal parameters, and *ω* = *π*/6 corresponds to a one-year period of time.

### 2.1. Model Assumptions

The following assumptions are considered in the formulation of the brucellosis model:

- Mixing of individuals in each population is homogeneous
- Infected animals shed *Brucella* in the environment
- Domestic and wild animals' seropositivity is lifelong
- Immunized livestock cannot be infected unless their resistance to infection wanes
- The natural mortality rate in each of the species is constant
- The birth rate for each population is greater than the natural mortality rate

The variables and parameter values per year incorporated in this model are summarized in Tables 1 and 2, respectively.

The interactions between humans, animals, and pathogens in the environment are shown in Figure 1, and the resulting model system is shown by equation (1).

(1) $$\begin{array}{c} \left\{\begin{array}{cc} \frac{dV_{\text{a}}}{dt} & =\phi S_{\text{a}}-\left(\psi +\mu_{\text{a}}\right)V_{\text{a}},\\ \frac{dS_{\text{a}}}{dt} & =\pi_{\text{a}}N_{\text{a}}+\psi V_{\text{a}}-\left(\beta_{\text{a}}\left(t\right)I_{\text{a}}+\alpha_{\text{a}}\left(t\right)B+\phi +\mu_{\text{a}}\right)S_{\text{a}},\\ \frac{dI_{\text{a}}}{dt} & =\left(\beta_{\text{a}}\left(t\right)I_{\text{a}}+\alpha_{\text{a}}\left(t\right)B\right)S_{\text{a}}-\left(\mu_{\text{a}}+d\right)I_{\text{a}},\\ \frac{dS_{\text{h}}}{dt} & =\pi_{\text{h}}N_{\text{h}}+\gamma R_{\text{h}}-\left(\beta_{\text{h}}\left(t\right)I_{\text{a}}+\beta_{\text{h}}I_{\text{h}}+\alpha_{\text{h}}\left(t\right)B+\mu_{\text{h}}\right)S_{\text{h}},\\ \frac{dI_{\text{h}}}{dt} & =\left(\beta_{\text{h}}\left(t\right)I_{\text{a}}+\alpha_{\text{h}}\left(t\right)B\right)S_{\text{h}}-\left(\sigma +\mu_{\text{h}}\right)I_{\text{h}},\\ \frac{dR_{\text{h}}}{dt} & =\sigma I_{\text{h}}-\left(\gamma +\mu_{\text{h}}\right)R_{\text{h}},\\ \frac{dS_{\text{w}}}{dt} & =\pi_{\text{w}}N_{\text{w}}-\left(\beta_{\text{w}}\left(t\right)I_{\text{w}}+\alpha_{\text{w}}\left(t\right)B+\mu_{\text{w}}\right)S_{\text{w}},\\ \frac{dI_{\text{w}}}{dt} & =\left(\beta_{\text{w}}I_{\text{w}}+\alpha_{\text{w}}\left(t\right)B\right)-\mu_{\text{w}}I_{\text{w}},\\ \frac{dB}{dt} & =\rho \left(t\right)I_{\text{a}}+\rho_{\text{w}}\left(t\right)I_{\text{w}}-\left(\tau +\varepsilon \left(t\right)\right)B. \end{array}\right. \end{array}$$

### 2.2. Model Properties

In this section, we use the box invariance method proposed by [40] to assess the well-posedness of the model (1) (existence and feasibility of its solution). In other words, we investigate whether the solutions of system (1) that have nonnegative initial values remain nonnegative for all times *t* ≥ 0. The compact form of system (1) can be expressed as

(2) $$\begin{array}{c} \frac{dX}{dt}=AX+F, \end{array}$$

where *X* = (*V*_a_, *S*_a_, *I*_a_, *S*_h_, *I*_h_, *R*_h_, *S*_w_, *I*_w_, *B*) and *F* is a column vector given by

(3) $$\begin{array}{c} F={\left(0,\pi_{c}N_{c},0,\pi_{\text{h}}N_{\text{h}},0,0,\pi_{\text{w}}N_{\text{w}},0,0\right)}^{T},\\ A=\left[\begin{array}{ccccccccc} -\left(\psi +\mu_{\text{a}}\right) & \phi & 0 & 0 & 0 & 0 & 0 & 0 & 0\\ \psi & -\lambda_{1} & 0 & 0 & 0 & 0 & 0 & 0 & 0\\ 0 & \lambda_{1} & -\left(\mu_{\text{a}}+d\left(t\right)\right) & 0 & 0 & 0 & 0 & 0 & 0\\ 0 & 0 & 0 & \lambda_{2}+\mu_{\text{h}} & 0 & \gamma & 0 & 0 & 0\\ 0 & 0 & 0 & \lambda_{1} & -\left(\sigma +\mu_{\text{h}}\right) & 0 & 0 & 0 & 0\\ 0 & 0 & 0 & 0 & \sigma & -\left(\gamma +\mu_{\text{h}}\right) & 0 & 0 & 0\\ 0 & 0 & 0 & 0 & 0 & 0 & -\left(\lambda_{3}+\mu_{\text{w}}\right) & 0 & 0\\ 0 & 0 & 0 & 0 & 0 & 0 & \lambda_{3} & -\mu_{\text{w}} & 0\\ 0 & 0 & \rho & 0 & 0 & 0 & 0 & \rho_{\text{w}} & -\lambda \end{array}\right], \end{array}$$

where

(4) $$\begin{array}{c} \lambda_{\text{a}}=\left(\beta_{\text{a}}\left(t\right)I_{\text{a}}+\alpha \left(t\right)B+\phi +\mu_{\text{a}}\right),\\ \lambda_{2}=\beta_{\text{h}}\left(t\right)I_{\text{a}}+\beta_{\text{h}}\left(t\right)I_{\text{h}}+\alpha_{\text{h}}B,\\ \lambda_{3}=\beta_{\text{w}}\left(t\right)I_{\text{w}}+\alpha_{\text{w}}\left(t\right)B,\\ \lambda =\left(\tau +\varepsilon \left(t\right)\right). \end{array}$$

It can be noticed that *A* is the Metzler matrix for all *X* ∈ ℝ_+_^9^. Therefore, based on the fact that *F* ≥ 0, model (1) is positively invariant in ℝ_+_^9^. This implies that an arbitrary trajectory of the system starting in ℝ_+_^9^ forever remains in ℝ_+_^9^. In addition, *F* is Lipschitz continuous. Thus, a unique maximal solution exists, and so

(5) $$\begin{array}{c} D=\left\{\left(V_{\text{a}},S_{\text{a}},I_{\text{a}},S_{\text{h}},I_{\text{h}},R_{\text{h}},S_{\text{w}},I_{\text{w}},B\right)\geq 0\right\}\in {\mathbb{R}}_{+}^{9} \end{array}$$

is the feasible region for the model (1). Thus, model (1) is epidemiologically and mathematically well-posed in the region *𝒟*.

### 2.3. Brucellosis-Free Equilibrium

The brucellosis-free equilibrium solution for system (1) is computed and found to be

(6) $$\begin{array}{c} \left(V_{\text{a}}^{0},S_{\text{a}}^{0},I_{\text{a}}^{0},S_{\text{h}}^{0},I_{\text{h}}^{0},R_{\text{h}}^{0},S_{\text{w}}^{0},I_{\text{w}}^{0},B^{0}\right)=\left(\frac{\phi \pi_{\text{a}}N_{\text{a}}}{\mu_{\text{a}}\left(\phi +\psi +\mu_{\text{a}}\right)},\frac{\left(\psi +\mu_{\text{a}}\right)\pi_{\text{a}}N_{\text{a}}}{\mu_{\text{a}}\left(\phi +\psi +\mu_{\text{a}}\right)},0,\frac{\pi_{\text{h}}N_{\text{h}}}{\mu_{\text{h}}},0,0,\frac{\pi_{\text{w}}N_{\text{w}}}{\mu_{\text{w}}},0,0\right), \end{array}$$

where *N*_a_, *N*_h_, and *N*_w_ are, respectively, the initial total populations of the livestock, humans, and wild animals.

### 2.4. The Reproduction Number

A heterogeneous population with individuals which can be grouped into *n* homogeneous compartments is considered in this section. Let *x* = (*x*_1_, ⋯,*x*_*n*_)^*T*^, with *x*_*i*_ ≥ 0, be the state of individuals in each compartment. It is assumed that the compartments can be divided into the following: infected designated as *i* = 1, ⋯, *m* and uninfected designated as *i* = *m* + 1, ⋯, *n*. We also define *X*_s_ to be the set of all disease-free states:

(7) $$\begin{array}{c} X_{\text{s}}=\left\{x\geq 0:x_{i}=0,\forall i=1,\cdots ,m\right\}. \end{array}$$

Let *ℱ*_*i*_(*t*, *x*) be the input rate of newly infected individuals in the *i*^th^ compartment, *𝒱*_*i*_^+^(*t*, *x*) be the input rate of individuals by other means (for example, births and immigrations), and *𝒱*_*i*_^−^(*t*, *x*) be the rate of transfer of individuals out of compartment *i* (for example, deaths, recovery, and emigrations). Henceforth, the disease transmission model is governed by a nonautonomous ordinary differential system:

(8) $$\begin{array}{c} \frac{dx_{i}}{dt}=F_{i}\left(t,x\right)-V_{i}\left(t,x\right)≜f_{i}\left(t,x\right),i=1,\cdots ,n, \end{array}$$

where *𝒱*_*i*_(*t*, *x*) = *𝒱*_*i*_^−^(*t*, *x*) − *𝒱*_*i*_^+^(*t*, *x*).

Succeeding the approach by [41] and that of [42] for epidemic models, we look at conditions (A1)–(A7) for the brucellosis model. The model (1) is equivalent to periodic ordinary differential system (8), we can easily see that conditions (A1)–(A5) stated below are satisfied.

(A1) For each 1 ≤ *i* ≤ *n*, the functions *ℱ*_*i*_(*t*, *x*), *𝒱*_*i*_^+^(*t*, *x*), and *𝒱*_*i*_^−^(*t*, *x*) are nonnegative and continuous on ℝ × ℝ_+_^*n*^ and continuously differential with respect to *x*. This is based on the fact that each function denotes a directed nonnegative transfer of individuals

(A2) There is a real number *ω* > 0 such that for each 1 ≤ *i* ≤ *n*, the functions *ℱ*_*i*_(*t*, *x*), *𝒱*_*i*_^+^(*t*, *x*), and *𝒱*_*i*_^−^(*t*, *x*) are *ω*-periodic in *t*. This biologically describes a periodic environment due to seasonality

(A3) If *x*_*i*_ = 0, then *𝒱*_*i*_^−^(*t*, *x*) = 0. In particular, if *x* ∈ *X*_s_, then *𝒱*_*i*_^−^(*t*, *x*) = 0 for *i* = 1, ⋯, *m*. That is, if a compartment is empty, then there is no transfer of individuals out of it

(A4) *ℱ*_*i*_ = 0 for *i* > *m*. This means that the infection incidence for uninfected compartments is zero

(A5) If *x* ∈ *X*_s_, then *ℱ*_*i*_ = *𝒱*_*i*_^+^ = 0 for *i* = 1, ⋯, *m*. This implies that if the population is disease-free in the beginning, it will remain so

We know that model (8) has a disease-free periodic solution, so we define a 5 × 5 matrix for the nontransmitting compartments as

(9) $$\begin{array}{c} M\left(t\right)=\left[\begin{array}{ccccc} -\left(\psi +\mu_{\text{a}}\right) & \phi & 0 & 0 & 0\\ \psi & -\left(\phi +\mu_{\text{a}}\right) & 0 & 0 & 0\\ 0 & 0 & -\mu_{\text{h}} & \gamma & 0\\ 0 & 0 & 0 & -\left(\gamma +\mu_{\text{h}}\right) & 0\\ 0 & 0 & 0 & 0 & -\mu_{\text{w}} \end{array}\right]. \end{array}$$

Let *Φ*_*M*_(*t*) be the monodromy matrix of the linear *ω*-periodic system *dz*/*dt* = *M*(*t*)*z*. Then, *ρ*(*Φ*_*M*_(*ω*)) < 1 implying that *E*^0^(*t*) is linearly asymptotically stable in the disease-free subspace *X*_s_; that is,

(A6) *ρ*(*Φ*_*M*_(*ω*)) < 1, where *ρ*(*Φ*_*M*_(*ω*)) is the spectral radius of *Φ*_*M*_(*ω*), is satisfied

For convenience purposes and easy presentation of the results, we let *C* denote all continuous functions on the real line. If *f* is a periodic function in *C*, then we use $\bar{f}$ for the average value of the time interval [0*T*] defined by

(10) $$\begin{array}{c} \bar{f}=\frac{1}{T}\int_{0}^{T}\;f\left(t\right)dt, \end{array}$$

for continuous *T* periodic function *f*(*t*). Inspired by the approach of [41, 43], we obtain

(11) $$\begin{array}{c} F=\left[\begin{array}{cccc} \frac{\left(\psi +\mu_{\text{a}}\right){\bar{\beta }}_{\text{a}}\left(t\right)\pi_{\text{a}}N_{\text{a}}}{\mu_{\text{a}}\left(\phi +\psi +\mu_{\text{a}}\right)} & 0 & 0 & \frac{\left(\psi +\mu_{\text{a}}\right){\bar{\alpha }}_{\text{a}}\left(t\right)\pi_{\text{a}}N_{\text{a}}}{\mu_{\text{a}}\left(\phi +\psi +\mu_{\text{a}}\right)}\\ \frac{{\bar{\beta }}_{\text{h}}\left(t\right)\pi_{\text{h}}N_{\text{h}}}{\mu_{\text{h}}} & \frac{{\bar{\beta }}_{\text{h}}\left(t\right)\pi_{\text{h}}N_{\text{h}}}{\mu_{\text{h}}} & 0 & \frac{{\bar{\alpha }}_{\text{h}}\left(t\right)\pi_{\text{h}}N_{\text{h}}}{\mu_{\text{h}}}\\ 0 & 0 & \frac{{\bar{\beta }}_{\text{w}}\left(t\right)\pi_{\text{w}}N_{\text{w}}}{\mu_{\text{w}}} & \frac{{\bar{\alpha }}_{\text{w}}\left(t\right)\pi_{\text{w}}N_{\text{w}}}{\mu_{\text{w}}}\\ {\bar{\rho }}_{\text{a}}\left(t\right) & 0 & {\bar{\rho }}_{\text{w}}\left(t\right) & 0 \end{array}\right], \end{array}$$

(12) $$\begin{array}{c} V=\left[\begin{array}{cccc} \mu_{\text{a}}+d & 0 & 0 & 0\\ 0 & \sigma +\mu_{\text{h}} & 0 & 0\\ 0 & 0 & \mu_{\omega } & 0\\ 0 & 0 & 0 & \left(\tau +\bar{\varepsilon }\left(t\right)\right) \end{array}\right] \end{array}$$

and observe that *F* is nonnegative and (−*V*) is cooperative because its off-diagonal elements are nonnegative.

It follows that the effective reproductive number of the time-averaged autonomous system is

(13) $$\begin{array}{c} \left[R_{e}\right]=\frac{R_{11}+R_{33}+\sqrt{{\left(R_{11}-R_{33}\right)}^{2}+4R_{13}R_{31}}}{2}, \end{array}$$

where

(14) $$\begin{array}{c} R_{11}=\frac{\left({\bar{\beta }}_{\text{a}}\left(t\right)\left(\tau +\bar{\varepsilon }\left(t\right)\right)+{\bar{\alpha }}_{\text{a}}\left(t\right)\bar{\rho }\left(t\right)\right)\left(\psi +\mu_{\text{a}}\right)\pi_{\text{a}}N_{\text{a}}}{\mu_{\text{a}}\left(\phi +\psi +\mu_{\text{a}}\right)\left(\mu_{\text{a}}+d\right)\left(\tau +\bar{\varepsilon }\left(t\right)\right)},\\ R_{33}=\frac{\left({\bar{\beta }}_{\text{w}}\left(t\right)\left(\tau +\bar{\varepsilon }\left(t\right)\right)+{\bar{\alpha }}_{\text{w}}\left(t\right){\bar{\rho }}_{\text{w}}\left(t\right)\right)\left(\psi +\mu_{\text{a}}\right)\pi_{\text{w}}N_{\text{w}}}{\mu_{\text{w}}^{2}\left(\tau +\bar{\varepsilon }\left(t\right)\right)},\\ R_{13}=\frac{{\bar{\alpha }}_{\text{a}}\left(t\right){\bar{\rho }}_{\text{w}}\left(t\right)\left(\psi +\mu_{\text{a}}\right)\pi_{\text{a}}N_{\text{a}}}{\mu_{\text{a}}\mu_{\text{w}}\left(\tau +\bar{\varepsilon }\left(t\right)\right)\left(\phi +\psi +\mu_{\text{a}}\right)},\\ R_{31}=\frac{{\bar{\alpha }}_{\text{w}}\left(t\right)\rho \left(t\right)\pi_{\text{w}}N_{\text{w}}}{\mu_{\text{w}}\left(\mu_{\text{a}}+d\right)\left(\tau +\bar{\varepsilon }\left(t\right)\right)}. \end{array}$$

Generally, the time-averaged effective reproduction number is computed as the dominant eigenvalue of *FV*^−1^ using the Maple package and is found to be

(15) $$\begin{array}{c} \rho \left(FV^{-1}\right)=\left[R_{e}\right]=\frac{1}{T}\int_{0}^{T}\;\frac{R_{11}+R_{33}+\sqrt{{\left(R_{11}-R_{33}\right)}^{2}+4R_{13}R_{31}}}{2}ds. \end{array}$$

If no interventions are administered, the time-averaged basic reproductive number for model system (1) is found to be

(16) $$\begin{array}{c} \left[R_{0}\right]=\frac{1}{T}\int_{0}^{T}\;\frac{R_{11}^{0}+R_{33}^{0}+\sqrt{{\left(R_{11}^{0}-R_{33}^{0}\right)}^{2}+4R_{13}^{0}R_{31}^{0}}}{2}ds, \end{array}$$

where

(17) $$\begin{array}{c} R_{11}=\frac{\left({\bar{\beta }}_{\text{a}}\left(t\right)\bar{\varepsilon }\left(t\right)+{\bar{\alpha }}_{\text{a}}\left(t\right)\bar{\rho }\left(t\right)\right)\pi_{\text{a}}N_{\text{a}}}{\mu_{\text{a}}^{2}\bar{\varepsilon }\left(t\right)},\\ R_{33}=\frac{\left({\bar{\beta }}_{\text{w}}\left(t\right)\bar{\varepsilon }\left(t\right)+{\bar{\alpha }}_{\text{w}}\left(t\right){\bar{\rho }}_{\text{w}}\left(t\right)\mu_{\text{a}}\right)\pi_{\text{w}}N_{\text{w}}}{\mu_{\text{w}}^{2}\bar{\varepsilon }\left(t\right)},\\ R_{13}=\frac{{\bar{\alpha }}_{\text{a}}\left(t\right){\bar{\rho }}_{\text{w}}\left(t\right)\pi_{\text{a}}N_{\text{a}}}{\mu_{\text{a}}\mu_{\text{w}}\bar{\varepsilon }\left(t\right)},\\ R_{31}=\frac{{\bar{\alpha }}_{\text{w}}\left(t\right)\rho \left(t\right)\pi_{\text{w}}N_{\text{w}}}{\mu_{\text{w}}\mu_{\text{a}}\bar{\varepsilon }\left(t\right)}. \end{array}$$

[*R*_0_] may be interpreted as the average number of secondary cases arising from the introduction of a single infected person into a completely susceptible population at a random time of the year. The condition [*R*_0_] < 1 is sufficient and necessary for long-term disease extinction. Furthermore, let *Y*(*t*, *s*), *t* ≥ *s*, be the evolution operator of the linear *ω*-periodic system:

(18) $$\begin{array}{c} \frac{dy}{dt}=-V\left(t\right)y. \end{array}$$

That is, for each *s* ∈ ℝ, the 4 × 4 matrix *Y*(*t*, *s*) satisfies

(19) $$\begin{array}{c} \frac{d}{dt}Y\left(t,s\right)=-V\left(t\right)Y\left(t,s\right),\;\forall t\geq s,Y\left(s,s\right)=I, \end{array}$$

where *I* is a 4 × 4 identity matrix. Therefore, the monodromy matrix *Φ*_*V*_(*t*) of (18) equals *Y*(*t*, 0), *t* ≥ 0. Thus, condition (A7) below is satisfied.

(A7) The internal evolution of individuals in the infectious compartments due to deaths and movements is dissipative and decays exponentially in many cases. This is because of loss of infective members from natural and disease-induced mortality. Thus, *ρ*(*Φ*_*V*_(*ω*)) < 1

Based on the assumptions (A1)–(A7), we are now able to analyze the reproduction ratios for the epidemic model system (1). For this purpose, we always assume that the population is near the disease-free periodic state *E*^0^(*t*). By the standard theory of linear periodic systems [44], there exist *K* > 0 and *α* > 0 such that

(20) $$\begin{array}{c} \left\|Y\left(t,s\right)\right\|\leq Ke^{-\alpha \left(t-s\right)},\;\forall t\geq s,s\in \mathbb{R}. \end{array}$$

Consequently,

(21) $$\begin{array}{c} \left\|Y\left(t,t-a\right)F\left(t-a\right)\right\|\leq K\left\|F\left(t-a\right)\right\|e^{-\alpha a},\;\forall t\in \mathbb{R},a\in \left[0,\infty \right). \end{array}$$

In the computation of the basic reproduction number for the nonautonomous model system (1), we follow the method by [42]. Suppose Γ(*s*) is the initial distribution of infectious individuals in this periodic environment; then, *F*(*s*)Γ(*s*) is the rate of new infectious individuals produced by the infected individuals who were introduced at time *s*. *Y*(*t*, *s*)*F*(*s*)Γ(*s*) represents the distribution of the newly infected at time *s* and remains in the infected compartment at time *t* ≥ *s*. It follows that the cumulative distribution of new infections at *t* produced by all infected Γ(*t*) individuals introduced prior to *t* = *s* is given by

(22) $$\begin{array}{c} \Psi \left(t\right)=\int_{-\infty }^{t}\;Y\left(t,s\right)F\left(s\right)\Gamma \left(s\right)ds=\int_{0}^{\infty }\;Y\left(t,t-a\right)F\left(t,t-a\right)\Gamma \left(t-a\right)da,\;\forall t\in \mathbb{R},\Gamma \in C_{\omega }. \end{array}$$

Let *C*_*ω*_ be the ordered Banach space of all *ω*-periodic functions from ℝ to ℝ^*n*^, which is equipped with the maximum norm, ‖.‖_∞_, and the positive cone *C*_*ω*_^+^ = {Γ ∈ *C*_*ω*_Γ(*t*) ≥ 0, *t* ∈ ℝ}. We define the linear operator *L* : *C*_*ω*_*C*_*ω*_ by

(23) $$\begin{array}{c} \left(L\Gamma \right)\left(t\right)=\int_{0}^{\infty }\;Y\left(t,t-a\right)F\left(t,t-a\right)\Gamma \left(t-a\right)da,\;\forall t\in \mathbb{R},\Gamma \in C_{\omega }, \end{array}$$

where *L* is the next infection operator. Then, the basic reproduction number is given by

(24) $$\begin{array}{c} R_{\omega }=\rho \left(L\right), \end{array}$$

where *ρ*(*L*) is the spectral radius of *L*. By direct calculation, the evolution operator *Y*(*t*, *s*) for the system (1) is found to be

(25) $$\begin{array}{c} Y\left(t,s\right)=\left[\begin{array}{cccc} e^{-\left(\mu_{\text{a}}+d\right)\left(t-s\right)} & 0 & 0 & 0\\ 0 & e^{-\left(\sigma +\mu_{\text{h}}\right)\left(t-s\right)} & 0 & 0\\ 0 & 0 & e^{-\mu_{\omega }\left(t-s\right)} & 0\\ 0 & 0 & 0 & \bar{Y}\left(t,s\right) \end{array}\right], \end{array}$$

with

(26) $$\begin{array}{c} \bar{Y}\left(t,s\right)=e^{-\left(\tau +\varepsilon_{0}\right)\left(t-s\right)+\left(6\varepsilon_{0}\varepsilon_{1}/\pi \right)\left(\cos\left(\pi t/6\right)-\cos\left(\pi s/6\right)\right)}. \end{array}$$

Motivated by [45], the next infection operator can be numerically evaluated as

(27) $$\begin{array}{c} \left(L\varphi \right)\left(t\right)=\int_{0}^{\infty }\;Y\left(t,t-a\right)F\left(t,t-a\right)\Gamma \left(t-a\right)da=\int_{0}^{\omega }\;G\left(t,a\right)\Gamma \left(t-a\right)da, \end{array}$$

where

(28) $$\begin{array}{c} G\left(t,s\right)\approx \overset{M}{\underset{k=0}{\sum }}\;Y\left(t,t-s-k\omega \right)F\left(t-s\right)\approx \overset{M}{\underset{k=0}{\sum }}\;\left[\begin{array}{cccc} m_{11} & 0 & 0 & m_{14}\\ m_{21} & m_{22} & 0 & m_{24}\\ 0 & 0 & m_{33} & m_{33}\\ m_{41} & 0 & m_{43} & 0 \end{array}\right], \end{array}$$

for positive integers *M* which are large enough, and

(29) $$\begin{array}{c} \left\{\begin{array}{c} m_{11}=\frac{\beta_{\text{a}}\left(t-s\right)\left(\psi +\mu_{\text{a}}\right)\pi_{\text{a}}N_{\text{a}}}{\mu_{\text{a}}\left(\phi +\psi +\mu_{\text{a}}\right)}e^{-\left(\mu_{\text{a}}+d\right)\left(t-s\right)},\\ m_{14}=\frac{\alpha_{\text{a}}\left(t-s\right)\left(\psi +\mu_{\text{a}}\right)\pi_{\text{a}}N_{\text{a}}}{\mu_{\text{a}}\left(\phi +\psi +\mu_{\text{a}}\right)}e^{-\left(\mu_{\text{a}}+d\right)\left(t-s\right)},\\ m_{21}=\frac{\beta_{\text{h}}\left(t-s\right)\pi_{\text{h}}N_{\text{h}}}{\mu_{\text{h}}}e^{-\left(\sigma +\mu_{\text{a}}\right)\left(t-s\right)},\\ m_{22}=\frac{\beta_{\text{h}}\left(t-s\right)\pi_{\text{h}}N_{\text{h}}}{\mu_{\text{h}}}e^{-\left(\sigma +\mu_{\text{a}}\right)\left(t-s\right)},\\ m_{24}=\frac{\alpha_{\text{h}}\left(t-s\right)\pi_{\text{h}}N_{\text{h}}}{\mu_{\text{h}}}e^{-\left(\sigma +\mu_{\text{a}}\right)\left(t-s\right)},\\ m_{33}=\frac{\beta_{\text{w}}\left(t-s\right)\pi_{\text{h}}N_{\text{h}}}{\mu_{\text{h}}}e^{-\omega \left(t-s\right)},\\ m_{34}=\frac{\alpha_{\text{w}}\left(t-s\right)\pi_{\text{w}}N_{\text{w}}}{\mu_{\text{w}}}e^{-\omega \left(t-s\right)},\\ m_{41}=\rho \left(t-s\right)e^{-\left(\tau +\varepsilon_{0}\right)\left(t-s\right)+\left(6\varepsilon_{0}\varepsilon_{1}/\pi \right)\left(\cos\left(\frac{\pi t}{6}\right)-\cos\left(\frac{\pi s}{6}\right)\right)},\\ m_{43}=\rho_{\text{w}}\left(t-s\right)e^{-\left(\tau +\varepsilon_{0}\right)\left(t-s\right)+\left(6\varepsilon_{0}\varepsilon_{1}/\pi \right)\left(\cos\left(\frac{\pi t}{6}\right)-\cos\left(\frac{\pi s}{6}\right)\right)}. \end{array}\right. \end{array}$$

### 2.5. Global Stability of the Brucellosis-Free Solution

In this section, we establish the conditions for global stability of a disease-free periodic solution.

**Theorem 1 .**

The disease-free solution of system (1) is globally asymptotically stable if the basic reproduction number in *𝒟* is less than one.

**Proof**

Consider the matrix function:

(30) $$\begin{array}{c} F\left(t\right)-V\left(t\right)=\left[\begin{array}{cccc} \beta_{\text{a}}\left(t\right)S_{\text{a}}^{0}-\left(\mu_{\text{a}}+d\right) & 0 & 0 & \alpha_{\text{a}}\left(t\right)S_{\text{a}}^{0}\\ \frac{\beta_{\text{h}}\left(t\right)\pi_{\text{h}}N_{\text{h}}^{0}}{\mu_{\text{h}}} & \beta_{\text{h}}\left(t\right)S_{\text{h}}^{0}-\left(\sigma +\mu_{\text{h}}\right) & 0 & \frac{\alpha_{\text{h}}\left(t\right)\pi_{\text{h}}N_{\text{h}}^{0}}{\mu_{\text{h}}}\\ 0 & 0 & \beta_{\text{w}}\left(t\right)S_{\text{w}}^{0}-\mu_{\text{w}} & \frac{\alpha_{\text{w}}\left(t\right)\pi_{\text{w}}N_{\text{w}}}{\mu_{\text{w}}}\\ \rho \left(t\right) & 0 & \rho_{\text{w}}\left(t\right) & -\left(\tau +\varepsilon \left(t\right)\right) \end{array}\right]. \end{array}$$

We verify that matrix function (30) is continuous, cooperative, irreducible, and *ω*-periodic. Let *Φ*_(*F* − *V*)(.)_(*t*) be the fundamental solution matrix of the linear ordinary differential system:

(31) $$\begin{array}{c} \dot{x}=\left[F\left(t\right)-V\left(t\right)\right]x, \end{array}$$

and *ρ*(*Φ*_(*F* − *V*)(.)_(*ω*)) be the dominant eigenvalue of *Φ*_(*F* − *V*)(.)_(*ω*). From Theorem 2.2 in [42], we have *R*_0_ < 1 if and only if *ρ*(*Φ*_(*F* − *V*)(.)_(*ω*)) < 1.

**Lemma 1 .**

Let *v* = 1/*ωlnρ*(*Φ*_(*F* − *V*)(.)_(*ω*)). Then, there exists a positive *ω*-periodic function *v*(*t*) such that *e*^*vt*^*v*(*t*) is a solution to equation (31).

From the nondisease transmitting equations of system (1), we obtain the following:

(32) $$\begin{array}{c} V_{\text{a}}\left(t\right)\leq \frac{\phi \pi_{\text{a}}N_{\text{a}}}{\mu_{\text{a}}\left(\phi +\psi +\mu_{\text{a}}\right)}≜V_{\text{a}}^{0},\\ S_{\text{a}}\left(t\right)\leq \frac{\left(\psi +\mu_{\text{a}}\right)\pi_{\text{a}}N_{\text{a}}}{\mu_{\text{a}}\left(\phi +\psi +\mu_{\text{a}}\right)}≜S_{\text{a}}^{0},\\ S_{\text{h}}\left(t\right)\leq \frac{\pi_{\text{h}}N_{\text{h}}}{\mu_{\text{h}}}≜S_{\text{h}}^{0},\\ S_{\omega }\left(t\right)\leq \frac{\pi_{\text{w}}N_{\text{w}}}{\mu_{\text{w}}}≜S_{\text{w}}^{0}. \end{array}$$

Again, from the infectious and recovered classes of system (1), we have the following:

(33) $$\begin{array}{c} \frac{d}{dt}\left[\begin{array}{c} I_{\text{a}}\left(t\right)\\ I_{\text{h}}\left(t\right)\\ I_{\text{w}}\left(t\right)\\ B\left(t\right) \end{array}\right]\leq \left(F-V\right)\left[\begin{array}{c} I_{\text{a}}\left(t\right)\\ I_{\text{h}}\left(t\right)\\ I_{\text{w}}\left(t\right)\\ B\left(t\right) \end{array}\right]. \end{array}$$

Based on Lemma 2, there exists *v*(*t*) such that $x\left(t\right)=\left({\bar{I}}_{\text{a}}\left(t\right),{\bar{I}}_{\text{h}}\left(t\right),{\bar{I}}_{\text{w}}\left(t\right),\bar{B}\left(t\right)\right)=v\left(t\right)e^{vt}$ is a solution to equation (31) with *v* = 1/*ωlnρ*(*Φ*_(*F* − *V*)(.)_).

Based on the fact that *R*_0_ < 1, we have *ρ*(*Φ*_(*F* − *V*)(.)_) < 1 and *v* < 0. Thus,

(34) $$\begin{array}{c} \left(I_{\text{a}}\left(t\right),I_{\text{h}}\left(t\right),I_{\text{w}}\left(t\right),B\left(t\right)\right)\leq \left({\bar{I}}_{\text{a}}\left(t\right),{\bar{I}}_{\text{h}}\left(t\right),{\bar{I}}_{\text{w}}\left(t\right),\bar{B}\left(t\right)\right), \end{array}$$

when *t* is very large which would imply that

(35) $$\begin{array}{c} \underset{t\to \infty }{\lim}I_{\text{a}}\left(t\right)=\underset{t\to \infty }{\lim}I_{\text{h}}\left(t\right)=\underset{t\to \infty }{\lim}I_{\text{w}}\left(t\right)=\underset{t\to \infty }{\lim}B\left(t\right)=0. \end{array}$$

Moreover, as *t*⟶∞, we have

(36) $$\begin{array}{c} \frac{d}{dt}\left(V_{\text{a}}+S_{\text{a}}\right)⟶\pi_{\text{a}}N_{\text{a}}-\mu_{\text{a}}\left(V_{\text{a}}+S_{\text{a}}\right), \end{array}$$

which implies

(37) $$\begin{array}{c} \frac{dV_{\text{a}}}{dt}⟶\phi \left(\frac{\pi_{\text{a}}N_{\text{a}}}{\mu_{\text{a}}}-V_{\text{a}}\right)-\left(\psi +\mu_{\text{a}}\right)V_{\text{a}}=\frac{\psi \pi_{\text{a}}N_{\text{a}}}{\mu_{\text{a}}}-\left(\phi +\psi +\mu_{\text{a}}\right)V_{\text{a}}, \end{array}$$

(38) $$\begin{array}{c} \text{or}\frac{\phi \pi_{\text{a}}N_{\text{a}}}{\mu_{\text{a}}\left(\phi +\psi +\mu_{\text{a}}\right)}=V_{\text{a}}^{0}, \end{array}$$

which leads to

(39) $$\begin{array}{c} S_{\text{a}}\left(t\right)⟶\frac{\pi_{\text{a}}N_{\text{a}}}{\mu_{\text{a}}}-V_{\text{a}}^{0}=\frac{\left(\psi +\mu_{\text{a}}\right)\pi_{\text{a}}N_{\text{a}}}{\mu_{\text{a}}\left(\pi +\psi +\mu_{\text{a}}\right)}=S_{\text{a}}^{0}. \end{array}$$

Again,

(40) $$\begin{array}{c} \frac{dS_{\text{h}}}{dt}⟶\pi_{\text{h}}N_{\text{h}}-\mu_{\text{h}}S_{\text{h}},\\ \frac{dS_{\text{w}}}{dt}⟶\pi_{\text{w}}N_{\text{w}}-\mu_{\text{w}}S_{\text{w}}, \end{array}$$

which gives

(41) $$\begin{array}{c} S_{\text{h}}^{0}=\frac{\pi_{\text{h}}N_{\text{h}}}{\mu_{\text{h}}},\\ S_{\text{w}}^{0}=\frac{\pi_{\text{w}}N_{\text{w}}}{\mu_{\text{w}}}. \end{array}$$

Therefore,

(42) $$\begin{array}{c} \underset{t\to \infty }{\lim}x\left(t\right)=\left(V_{\text{a}}^{0},S_{\text{a}}^{0},0,S_{\text{h}}^{0},0,0,S_{\text{w}}^{0},0,0\right), \end{array}$$

for each solution *x*(*t*) in system (1).

### 2.6. Endemic Equilibrium Solution

This section is aimed at investigating the behavior of model system (1) when *R*_0_ > 1. We show that if *R*_0_ > 1, brucellosis infection persists in the animal and human populations and there exists a positive periodic solution. Following the approach in [46, 47], we define

(43) $$\begin{array}{c} X={\mathbb{R}}_{+}^{9};X_{0}={\mathbb{R}}_{+}^{4}\times \text{Int}{\left({\mathbb{R}}_{+}\right)}^{5};\partial X_{0}=X\backslash X_{0}. \end{array}$$

Let *L* : *𝒳*⟶*𝒳* be the Poncaré map associated with model system (1) such that *𝒫*(*x*_0_) = *u*(*ω*, *x*_0_)∀ *x*_0_ ∈ *𝒳*, where *u*(*t*, *x*_0_) denotes a unique solution of the system with *u*(0, *x*_0_) = *x*_0_.

**Definition 1 .**

The solutions of the model system (1) are said to be uniformly persistent if there exists some *ξ* > 0 such that

(44) $$\begin{array}{c} \underset{t\to \infty }{\lim}\text{Inf}V_{\text{a}}\left(t\right)>\xi ,\underset{t\to \infty }{\lim}\text{Inf}S_{\text{a}}\left(t\right)>\xi ,\underset{t\to \infty }{\lim}\text{Inf}I_{\text{a}}\left(t\right)>\xi ,\\ \underset{t\to \infty }{\lim}\text{Inf}S_{\text{h}}\left(t\right)>\xi ,\underset{t\to \infty }{\lim}\text{Inf}I_{\text{h}}\left(t\right)>\xi ,\underset{t\to \infty }{\lim}\text{Inf}R_{\text{h}}\left(t\right)>\xi ,\\ \underset{t\to \infty }{\lim}\text{Inf}S_{\text{w}}\left(t\right)>\xi ,\underset{t\to \infty }{\lim}\text{Inf}I_{\text{w}}\left(t\right)>\xi ,\underset{t\to \infty }{\lim}\text{Inf}B\left(t\right)>\xi , \end{array}$$

whenever

(45) $$\begin{array}{c} V_{\text{a}}\left(0\right)>0,S_{\text{a}}\left(0\right)>0,I_{\text{a}}\left(0\right)>0,S_{\text{h}}\left(0\right)>0,I_{\text{h}}\left(0\right)>0,R_{\text{h}}\left(0\right)>0,S_{\text{w}}\left(0\right)>0,I_{\text{w}}\left(0\right)>0,B\left(0\right)>0. \end{array}$$

**Theorem 2 .**

The solutions of the model system (1) are uniformly persistent, and the system admits at least one positive *ω*-periodic solution if *R*_0_ > 1.

**Proof**

We define

(46) $$\begin{array}{c} H_{\partial }=\left\{\left(V_{\text{a}}\left(0\right),S_{\text{a}}\left(0\right),I_{\text{a}}\left(0\right),S_{\text{h}}\left(0\right),I_{\text{h}}\left(0\right),R_{\text{h}}\left(0\right),S_{\text{w}}\left(0\right),I_{\text{w}}\left(0\right),B\left(0\right)\right)\in \partial X_{0}:P^{m}\left(V_{\text{a}}\left(0\right),S_{\text{a}}\left(0\right),I_{\text{a}}\left(0\right),S_{\text{h}}\left(0\right),I_{\text{h}}\left(0\right),R_{\text{h}}\left(0\right),S_{\text{w}}\left(0\right),I_{\text{w}}\left(0\right),B\left(0\right)\right)\in \partial X_{0},\;\forall m\geq 0\right\},\\ \tilde{H}=\left\{\left(V_{\text{a}}\left(0\right),S_{\text{a}}\left(0\right),0,S_{\text{h}}\left(0\right),0,0,S_{\text{w}}\left(0\right),0,0\right)\text{: }V_{\text{a}}\left(0\right)\geq 0,S_{\text{a}}\left(0\right)\geq 0,S_{\text{h}}\left(0\right)\geq 0,S_{\text{w}}\left(0\right)\geq 0\right\}. \end{array}$$

It is evident that ${\tilde{H}}_{\partial }\subseteq H_{\partial }$.

We first show that $H_{\partial }={\tilde{H}}_{\partial }.$ Consider the initial values:

(47) $$\begin{array}{c} \left(V_{\text{a}}\left(0\right),S_{\text{a}}\left(0\right),I_{\text{a}}\left(0\right),S_{\text{h}}\left(0\right),I_{\text{h}}\left(0\right),R_{\text{h}}\left(0\right),S_{\text{w}}\left(0\right),I_{\text{w}}\left(0\right),B\left(0\right)\right)\in \partial X_{0}\tilde{H}. \end{array}$$

If *I*_a_(0) = 0, *I*_h_(0), *I*_w_(0) = 0, and *B*(0) > 0, then based on the fact that there is a recruitment rate for susceptible individuals, we have *I*_a′_ > 0. Similarly, if *I*_w_(0) = 0, *I*_h_(0), *B*(0) = 0, and *I*_a_(0) > 0, then *B*′(0) > 0, *I*_a_(0) = 0, *I*_h_(0), *I*_w_(0) = 0, and *B*(0) > 0, and if *I*_a_(0) = 0, *I*_h_(0), *B*(0) = 0, and *I*_w_(0) > 0, then *B*′(0) > 0. It follows that (*V*_a_(*t*), *S*_a_(*t*), *I*_a_(*t*), *S*_h_(*t*), *I*_h_(*t*), *R*_h_(*t*), *S*_w_(*t*), *I*_w_(*t*), *B*(*t*)) ∉ *∂𝒳*_0_ for 0 < *t* ≪ 1. The positive invariance of *X*_0_ implies that $H_{\partial }={\tilde{H}}_{\partial }$.

Again, if we consider the fixed point:

(48) $$\begin{array}{c} H_{0}=\left(\frac{\phi \pi_{\text{a}}N_{\text{a}}}{\mu_{\text{a}}\left(\phi +\psi +\mu_{\text{a}}\right)},\frac{\left(\psi +\mu_{\text{a}}\right)\pi_{\text{a}}N_{\text{a}}}{\mu_{\text{a}}\left(\phi +\psi +\mu_{\text{a}}\right)},0,\frac{\pi_{\text{h}}N_{\text{h}}}{\mu_{\text{h}}},0,\frac{\pi_{\text{w}}N_{\text{w}}}{\mu_{\text{w}}},0,0\right), \end{array}$$

we define

(49) $$\begin{array}{c} W^{S}\left(H_{0}\right)=\left\{x_{0}:L^{m}\left(x_{0}\right)⟶H_{0},x⟶\infty \right\}. \end{array}$$

It can be deduced from system (1) that if *I*_a_ = *I*_h_ = *I*_w_ = *B* = 0 and *t*⟶∞,

(50) $$\begin{array}{c} V_{\text{a}}\left(t\right)⟶V_{\text{a}}^{0}=\frac{\phi \pi_{\text{a}}N_{\text{a}}}{\mu_{\text{a}}\left(\phi +\psi +\mu_{\text{a}}\right)},\\ S_{\text{a}}\left(t\right)⟶S_{a}^{0}\frac{\left(\psi +\mu_{\text{a}}\right)\pi_{\text{a}}N_{\text{a}}}{\mu_{\text{a}}\left(\phi +\psi +\mu_{\text{a}}\right)},\\ S_{\text{h}}\left(t\right)⟶S_{\text{h}}^{0}=\frac{\pi_{\text{h}}N_{\text{h}}}{\mu_{\text{h}}},\\ S_{\text{w}}\left(t\right)⟶S_{\text{w}}^{0}=\frac{\pi_{\text{w}}N_{\text{w}}}{\mu_{\text{w}}}. \end{array}$$

We prove that *W*^*S*^(*H*_0_)∩*𝒳*_0_ = ∅.

Let ‖.‖ denote a norm on ℝ_+_^9^. Based on the continuity of solutions with respect to the initial conditions, for every *ε* > 0, there exists *δ* > 0 but small such that for all

(51) $$\begin{array}{c} \left(V_{\text{a}}\left(0\right),S_{\text{a}}\left(0\right),I_{\text{a}}\left(0\right),S_{\text{h}}\left(0\right),I_{\text{h}}\left(0\right),R_{\text{h}}\left(0\right),S_{\text{w}}\left(0\right),I_{\text{w}}\left(0\right),B\left(0\right)\right)\in \partial X_{0}, \end{array}$$

with

(52) $$\begin{array}{c} \left\|\left(V_{\text{a}}\left(0\right),S_{\text{a}}\left(0\right),I_{\text{a}}\left(0\right),S_{\text{h}}\left(0\right),I_{\text{h}}\left(0\right),R_{\text{h}}\left(0\right),S_{\text{w}}\left(0\right),I_{\text{w}}\left(0\right),B\left(0\right)\right)-H_{0}\right\|\leq \delta , \end{array}$$

we have

(53) $$\begin{array}{c} \left\|u\left(t,\left(V_{\text{a}}\left(0\right),S_{\text{a}}\left(0\right),I_{\text{a}}\left(0\right),S_{\text{h}}\left(0\right),I_{\text{h}}\left(0\right),R_{\text{h}}\left(0\right),S_{\text{w}}\left(0\right),I_{\text{w}}\left(0\right),B\left(0\right)\right)\right)-u\left(t,H_{0}\right)\right\|\leq \varepsilon ,\;\forall t\in \left[0,\omega \right]. \end{array}$$

So we claim that

(54) $$\begin{array}{c} \underset{t\to \infty }{\lim}\sup\left\|\left(V_{\text{a}}\left(0\right),S_{\text{a}}\left(0\right),I_{\text{a}}\left(0\right),S_{\text{h}}\left(0\right),I_{\text{h}}\left(0\right),R_{\text{h}}\left(0\right),S_{\text{w}}\left(0\right),I_{\text{w}}\left(0\right),B\left(0\right)\right)-H_{0}\right\|\geq \delta ,\;\forall \left(V_{\text{a}}\left(0\right),S_{\text{a}}\left(0\right),I_{\text{a}}\left(0\right),S_{\text{h}}\left(0\right),I_{\text{h}}\left(0\right),R_{\text{h}}\left(0\right),S_{\text{w}}\left(0\right),I_{\text{w}}\left(0\right),B\left(0\right)\right)\in X_{0} \end{array}$$

and prove by contradiction as follows:

Suppose

(55) $$\begin{array}{c} \underset{t\to \infty }{\lim}\sup\left\|\left(V_{\text{a}}\left(0\right),S_{\text{a}}\left(0\right),I_{\text{a}}\left(0\right),S_{\text{h}}\left(0\right),I_{\text{h}}\left(0\right),R_{\text{h}}\left(0\right),S_{\text{w}}\left(0\right),I_{\text{w}}\left(0\right),B\left(0\right)\right)-H_{0}\right\|<\delta , \end{array}$$

for some

(56) $$\begin{array}{c} \left(V_{\text{a}}\left(0\right),S_{\text{a}}\left(0\right),I_{\text{a}}\left(0\right),S_{\text{h}}\left(0\right),I_{\text{h}}\left(0\right),R_{\text{h}}\left(0\right),S_{\text{w}}\left(0\right),I_{\text{w}}\left(0\right),B\left(0\right)\right)\in X_{0}. \end{array}$$

In addition, we assume without loss of generality that

(57) $$\begin{array}{c} P^{m}\left\|\left(V_{\text{a}}\left(0\right),S_{\text{a}}\left(0\right),I_{\text{a}}\left(0\right),S_{\text{h}}\left(0\right),I_{\text{h}}\left(0\right),R_{\text{h}}\left(0\right),S_{\text{w}}\left(0\right),I_{\text{w}}\left(0\right),B\left(0\right)\right)-H_{0}\right\|<\delta ,\;\forall m\geq 0. \end{array}$$

Therefore, ∀*t* ∈ [0, *ω*], *m* ≥ 0, we have

(58) $$\begin{array}{c} \left\|u\left(t,\left(V_{\text{a}}\left(0\right),S_{\text{a}}\left(0\right),I_{\text{a}}\left(0\right),S_{\text{h}}\left(0\right),I_{\text{h}}\left(0\right),R_{\text{h}}\left(0\right),S_{\text{w}}\left(0\right),I_{\text{w}}\left(0\right),B\left(0\right)\right)\right)-u\left(t,H_{0}\right)\right\|\leq \varepsilon . \end{array}$$

Furthermore, for any nonnegative *t*, we can write *t* = *t*_0_ + *nω* with *t*_0_ ∈ [0, *ω*] and *n* being the greatest integer less than or equal to *t*/*ω*. Then, we get

(59) $$\begin{array}{c} \left\|u\left(t,\left(V_{\text{a}}\left(0\right),S_{\text{a}}\left(0\right),I_{\text{a}}\left(0\right),S_{\text{h}}\left(0\right),I_{\text{h}}\left(0\right),R_{\text{h}}\left(0\right),S_{\text{w}}\left(0\right),I_{\text{w}}\left(0\right),B\left(0\right)\right)\right)-u\left(t,H_{0}\right)\right\|=\left\|u\left(t_{0},\left(V_{\text{a}}\left(0\right),S_{\text{a}}\left(0\right),I_{\text{a}}\left(0\right),S_{\text{h}}\left(0\right),I_{\text{h}}\left(0\right),R_{\text{h}}\left(0\right),S_{\text{w}}\left(0\right),I_{\text{w}}\left(0\right),B\left(0\right)\right)\right)-u\left(t_{0},H_{0}\right)\right\|\leq \varepsilon , \end{array}$$

for any *t* > 0.

Let

(60) $$\begin{array}{c} \left(V_{\text{a}}\left(t\right),S_{\text{a}}\left(t\right),I_{\text{a}}\left(t\right),S_{\text{h}}\left(t\right),I_{\text{h}}\left(t\right),R_{\text{h}}\left(t\right),S_{\text{w}}\left(t\right),I_{\text{w}}\left(t\right),B\left(t\right)\right)=\left(V_{\text{a}}\left(0\right),S_{\text{a}}\left(0\right),I_{\text{a}}\left(0\right),S_{\text{h}}\left(0\right),I_{\text{h}}\left(0\right),R_{\text{h}}\left(0\right),S_{\text{w}}\left(0\right),I_{\text{w}}\left(0\right),B\left(0\right)\right). \end{array}$$

It follows that

(61) $$\begin{array}{c} \frac{\phi \pi_{\text{a}}N_{\text{a}}}{\mu_{\text{a}}\left(\phi +\psi +\mu_{\text{a}}\right)}-\varepsilon <V_{\text{a}}\left(t\right)<\frac{\phi \pi_{\text{a}}N_{\text{a}}}{\mu_{\text{a}}\left(\phi +\psi +\mu_{\text{a}}\right)}+\varepsilon ,\frac{\left(\psi +\mu_{a}\right)\pi_{\text{a}}N_{\text{a}}}{\mu_{\text{a}}\left(\phi +\psi +\mu_{\text{a}}\right)}-\varepsilon <S_{\text{a}}\left(t\right)<\frac{\left(\psi +\mu_{\text{a}}\right)\pi_{\text{a}}N_{\text{a}}}{\mu_{\text{a}}\left(\phi +\psi +\mu_{\text{a}}\right)}+\varepsilon ,\frac{\pi_{\text{h}}N_{\text{h}}}{\mu_{\text{h}}}-\varepsilon <S_{\text{h}}\left(t\right)<\frac{\pi_{\text{h}}N_{\text{h}}}{\mu_{\text{h}}},\frac{\pi_{\text{w}}N_{\text{w}}}{\mu_{\text{w}}}-\varepsilon <S_{\text{w}}\left(t\right)<\frac{\pi_{\text{w}}N_{\text{w}}}{\mu_{\text{w}}},0<I_{\text{a}}\left(t\right)<\varepsilon ,0<I_{\text{h}}\left(t\right)<\varepsilon ,0<I_{\text{w}}\left(t\right)<\varepsilon ,0<B\left(t\right)<\varepsilon . \end{array}$$

Then, we have

(62) $$\begin{array}{c} \frac{dI_{\text{a}}}{dt}=\left(\beta_{1}\left(t\right)I_{\text{a}}+\alpha_{1}\left(t\right)B\right)S_{\text{a}}-\left(\mu_{\text{a}}+d\right)I_{\text{a}}\geq \left(\beta_{1}\left(t\right)I_{\text{a}}+\alpha_{1}\left(t\right)B\right)\left(\frac{\left(\psi +\mu_{\text{a}}\right)\pi_{\text{a}}N_{\text{a}}}{\mu_{\text{a}}\left(\phi +\psi +\mu_{\text{a}}\right)}-\varepsilon \right)-\left(\mu_{\text{a}}+d\right)I_{\text{a}}=\left(\beta_{1}\left(t\right)I_{\text{a}}+\alpha_{1}\left(t\right)B\right)\left(\frac{\left(\psi +\mu_{\text{a}}\right)\pi_{\text{a}}N_{\text{a}}}{\mu_{\text{a}}\left(\phi +\psi +\mu_{\text{a}}\right)}\right)-\left(\mu_{\text{a}}+d\right)I_{\text{a}}-\varepsilon \left(\beta_{1}\left(t\right)I_{\text{a}}+\alpha_{1}\left(t\right)B\right). \end{array}$$

Similarly,

(63) $$\begin{array}{c} \frac{dI_{\text{h}}}{dt}\geq \left(\beta_{2}\left(t\right)I_{\text{h}}+\alpha_{2}\left(t\right)B\right)\left(\frac{\pi_{\text{h}}N_{\text{h}}}{\mu_{\text{h}}}\right)-\left(\sigma +\mu_{\text{h}}\right)I_{\text{h}}-\varepsilon \left(\beta_{2}\left(t\right)I_{\text{h}}+\alpha_{2}\left(t\right)B\right),\\ \frac{dI_{\text{w}}}{dt}\geq \left(\beta_{\text{w}}\left(t\right)I_{\text{w}}+\alpha_{\text{w}}\left(t\right)B\right)\left(\frac{\pi_{\text{w}}N_{\text{w}}}{\mu_{\text{w}}}\right)-\mu_{\text{w}}I_{\text{w}}-\varepsilon \left(\beta_{\text{w}}\left(t\right)I_{\text{w}}+\alpha_{\text{w}}\left(t\right)B\right). \end{array}$$

Thus, we obtain

(64) $$\begin{array}{c} \frac{d}{dt}\left[\begin{array}{c} I_{\text{a}}\left(t\right)\\ I_{\text{h}}\left(t\right)\\ I_{\text{w}}\left(t\right)\\ B\left(t\right) \end{array}\right]\geq \left(F-V-\varepsilon K\right)\left[\begin{array}{c} I_{\text{a}}\left(t\right)\\ I_{\text{h}}\left(t\right)\\ I_{\text{w}}\left(t\right)\\ B\left(t\right) \end{array}\right]. \end{array}$$

But *R*_0_ > 1 if and only if *ρ*(*Φ*_(*F* − *V*)(.)_) > 1. Thus, for *ε* > 0 whenever small, we have *ρ*(*Φ*_(*F* − *V*)(.)_) > 1. Using Lemma 2 and the comparison principle, we get

(65) $$\begin{array}{c} \underset{t\to \infty }{\lim}I_{\text{a}}\left(t\right)=\underset{t\to \infty }{\lim}I_{\text{h}}\left(t\right)=\underset{t\to \infty }{\lim}I_{\text{w}}\left(t\right)=\underset{t\to \infty }{\lim}B\left(t\right)=\infty , \end{array}$$

which contradicts our original assumption.

Thus, *H*_0_ is acyclic in *H*_*∂*_, and *𝒫* is uniformly persistent with respect to (*𝒳*_0_, *∂𝒳*_0_), which implies the uniform persistence of the solutions to the original system [47]. Consequently, the Poincaré map *p* has a fixed point:

(66) $$\begin{array}{c} \left({\bar{V}}_{\text{a}}\left(0\right),{\bar{S}}_{\text{a}}\left(0\right),{\bar{I}}_{\text{a}}\left(0\right),{\bar{S}}_{\text{h}}\left(0\right),{\bar{I}}_{\text{h}}\left(0\right),{\bar{S}}_{\text{w}}\left(0\right),{\bar{I}}_{\text{w}}\left(0\right),\bar{B}\left(0\right)\right)\in X_{0}, \end{array}$$

with *V*_a_(0), *S*_a_(0), *S*_h_(0), *S*_w_(0) ≠ 0. Thus,

(67) $$\begin{array}{c} \left({\bar{V}}_{\text{a}}\left(0\right),{\bar{S}}_{\text{a}}\left(0\right),{\bar{I}}_{\text{a}}\left(0\right),{\bar{S}}_{\text{h}}\left(0\right),{\bar{I}}_{\text{h}}\left(0\right),{\bar{S}}_{\text{w}}\left(0\right),{\bar{I}}_{\text{w}}\left(0\right),\bar{B}\left(0\right)\right)\in \text{Int}{\left({\mathbb{R}}_{+}\right)}^{9}, \end{array}$$

and

(68) $$\begin{array}{c} \left({\tilde{V}}_{\text{a}}\left(0\right),{\tilde{S}}_{\text{a}}\left(0\right),{\tilde{I}}_{\text{a}}\left(0\right),{\tilde{S}}_{\text{h}}\left(0\right),{\tilde{I}}_{\text{h}}\left(0\right),{\tilde{S}}_{\text{w}}\left(0\right),{\bar{I}}_{\text{w}}\left(0\right),\tilde{B}\left(0\right)\right)=u\left(t,\left({\tilde{V}}_{\text{a}}\left(0\right),{\tilde{S}}_{\text{a}}\left(0\right),{\tilde{I}}_{\text{a}}\left(0\right),{\tilde{S}}_{\text{h}}\left(0\right),{\tilde{I}}_{\text{h}}\left(0\right),{\tilde{S}}_{\text{w}}\left(0\right),{\bar{I}}_{\text{w}}\left(0\right),\tilde{B}\left(0\right)\right)\right) \end{array}$$

is a positive *ω*-periodic solution of the system.

## 3. Numerical Simulations

In this part, we perform numerical simulations for model system (1) for the purpose of verifying some of the analytical findings. The baseline parameter values used in our computations are mainly from literature similar to this work, and unavailable parameter values are assumed for illustration. The parameter descriptions and values per year are shown in Table 2. Figures 2–5 illustrate the variations in human, wild animal, and livestock subpopulations while Figure 6 shows the existence of a globally stable disease-free periodic solution. Additionally, Figures 7–9 highlight the impact of temperature variations on the transmission dynamics of brucellosis.  Figure 2 shows that the number of infective livestock decreases seasonally with an increase in time while Figure 2(a) illustrates a decrease in the susceptible animal subpopulation as time increases. The decrease in the number of infective livestock is due to proper implementation of vaccination and gradual culling of seropositive animals as control strategies. On the other hand, the sharp decrease in the susceptible animal subpopulation can be associated with the large number of infective animals and consequently high transmission rate in less than a one-year period of time while the gradual decrease in the next two years is due to vaccination programmes and decreased infection rate.  Figure 3 shows a strong relationship between the number of infective and susceptible humans. For instance, at *t* = 0, *S*_a_ = 5000 and *I*_a_ = 0 while at *t* = 3, *S*_a_ = 2555 and *I*_a_ = 1850. The seasonal increase in the individuals in Figure 3(a) is associated with the low human treatment rate and poor control of the disease from infective livestock as well as contaminated environment. Besides, the decrease in the number of susceptible humans in Figure 3(b) is due to the high transmission rate from both infective animals and their products while the increase may be associated with proper implementation of the control strategies such as environmental hygiene, animal vaccination, and gradual culling of seropositive animals [24].  Figure 4 shows that the number of susceptible wild animals decreases with the increase in infective wild animals. In particular, the introduction of 200 susceptible wild animals in the contaminated environment produces more than 200 infective wild animals. This is based on the fact that both infective and susceptible animals have free movements and interactions within their parks. Besides, lack of wild animal brucellosis control measures and the fact that the disease does not kill keep the number of infected wild animals seasonally increasing. This implies that, in order to control the transmission dynamics of brucellosis in livestock and humans, interactions between domestic and wild animals should be restricted.  Figure 5(a) shows that the number of *Brucella* bacteria in the environment decreases seasonally as the time increases while Figure 5(b) illustrates the variations in the number of recovered humans with respect to increase in time. These variations are associated with the regular implementation of the control strategies like environment hygiene and sanitation, human treatment, and gradual culling of infective animals. Furthermore, the recovered human population in the first six years increases due to effective treatment of the infective animals, and its decrease is associated with the decrease in the number of infected humans as well as proper control of the disease from livestock and their products. Figure 6 shows the existence of a stable periodic solution between the animal subpopulations and the number of *Brucella* bacteria in the environment.  Figure 7(a) shows the seasonal variations in the effective reproductive number with respect to maximum daily temperature while Figure 7(b) illustrates the changes in the effective reproduction number with respect to seasonal variations in minimum daily temperature.  Figure 8(a) illustrates the variations in the effective reproduction number versus maximum daily temperature while Figure 8(b) depicts the changes in the effective reproduction number with respect to seasonal variations in minimum daily temperature.  Figure 9 presents the comparison between direct and indirect routes of brucellosis transmission. In particular, high strength of seasonal forcing shown in Figure 9(a) is due to seasonality in both direct and indirect routes of disease transmission while the curve with low amplitude shows the impact of lack of seasonality on the direct disease transmission. Moreover, Figure 9(b) indicates that seasonality in direct transmission has a significant contribution to the brucellosis transmission than that in indirect transmission; the graph in red is for seasonality in both direct and indirect transmission while the one in blue is for seasonality in both.

Generally, findings from this study advocate that, when the weather condition favours the increase in the transmission rates of brucellosis in livestock, humans, wild animals, and the environment, the incidence of the disease increases significantly and vice versa. This implies that in order to effectively prevent, control, eliminate, or eradicate brucellosis from the community, measures should be timely taken in accordance with the fluctuation in the disease transmission rates as a result of daily temperature variations. Thus, to avoid underestimation or overestimation of the resources when dealing with brucellosis, the aspect of seasonal weather variation should be taken into account when planning for prevention, control, elimination, or eradication of brucellosis infections.

## Figures and Tables

**Figure 1:** Flow diagram for brucellosis dynamics in animals, environment, and humans.

**Figure 2:** Seasonal variations in the number of infective and susceptible animals.

**Figure 3:** Seasonal variations in the number of infective and susceptible humans.

**Figure 4:** Seasonal variations in the number of infective and susceptible wild animals.

**Figure 5:** Variations in the effective reproduction number with respect to changes in environmental hygiene and human treatment.

**Figure 6:** Relationship between *Brucella* spp. and susceptible and infected subpopulations.

**Figure 7:** Variations in the effective reproduction number with seasonal changes in temperature for the year 1979 in Mpwapwa District, Dodoma.

**Figure 8:** Variations in the effective reproduction number with seasonal changes in temperature for the year 2014 in Ngorongoro District, Arusha.

**Figure 9:** Variations in the effective reproduction number with seasonal changes in temperature for the year 2014 in Ngorongoro District, Arusha.

**Table 1:** Model variables.

Variable	Description
*S*_h_(*t*)	Number of susceptible humans at time *t*
*I*_h_(*t*)	Number of infected humans at time *t*
*R*_h_(*t*)	Number of recovered humans at time *t*
*S*_a_(*t*)	Number of susceptible animals at time *t*
*I*_a_(*t*)	Number of infected animals at time *t*
*V*_a_(*t*)	Number of vaccinated animals at time *t*
*B*(*t*)	Number of *Brucella* load per unit volume in the environment at time *t*

**Table 2:** Parameters of the model and their description.

Parameter	Description	Value	Source
*π*_a_	Per-capita livestock birth rate	0.1	[37]
*ϕ*_a_	Livestock vaccination rate	0.7	[37]
*π*_h_	Per-capita human birth rate	0.02	[38]
*σ*	Human recovery rate	0.25	[37]
*μ*_h_	Per-capita human natural death rate	0.02	[38]
*ψ*	Livestock vaccine efficacy waning rate	0.4	[31]
*β*_a_	Within-livestock transmission rate	0.0011	[31]
*d*	Gradual culling of seropositive livestock	0.35	[31]
*μ*_a_	Per-capita livestock natural mortality rate	0.25	[31]
*π*_w_	Per-capita wild animal birth rate	0.08	[39]
*β*_w_	Within-wild animal transmission rate	0.05	[39]
*α*_w_	*Brucella* from B to wild animal transmission rate	0.00035	[3]
*μ*_w_	Per-capita natural death rate of wild animals	0.07	[39]
*α*	*Brucella* from B to livestock transmission rate	0.00035	[3]
*α*_h_	*Brucella* from B to human transmission rate	0.002	[37]
*ρ*	*Brucella* shedding rate of infected livestock	0.5	[37]
*ρ*_w_	*Brucella* shedding rate of infected wild animals	15	[30]
*β*_h_	Livestock to human transmission rate	0.0002	[37]
*ε*	Decaying rate of *Brucella* in the environment	8	[31]
*τ*	Environmental hygiene and sanitation rate	12	[3]

## Data Availability

The data supporting the findings in the article were derived as follows: We used the set of parameter values mainly from articles similar to this work, while unavailable data, especially values of parameters, were estimated for the purpose of verifying results of the mathematical analyses of the models developed in the manuscript.
